# The Diagnosis of Early Gastric Cancer Based on Medical Imaging Technology and Mathematical Modeling

**DOI:** 10.1155/2022/8721654

**Published:** 2022-10-03

**Authors:** Jingying Xiu, Lie Ma, Yanping Ding, Yang Li, Lili Kan, Shi Feng, Fei Wu, Shanshan Xu, Xinan Lu, Ting He, Zhihai Han

**Affiliations:** ^1^Beijing Tongren Hospital, Capital Medical University, 100730 Beijing, China; ^2^Department of Pulmonary and Critical Care Medicine, The Sixth Medical Center of PLA General Hospital, 100048 Beijing, China; ^3^ImmunoChina Pharmaceuticals Co., Ltd., 100195 Beijing, China; ^4^Department of Pharmacy, Panjin Gem Flower Hospital, 124010 Panjin, Liaoning, China

## Abstract

The key to reducing the mortality of gastric cancer is early detection, early diagnosis, and early treatment of gastric cancer. Early diagnosis of gastric cancer is the key to early detection and diagnosis of gastric cancer. Early diagnosis and treatment of gastric cancer is of great significance for improving the curative effect and reducing mortality of gastric cancer. The purpose of this paper is to study the diagnosis of early gastric cancer based on medical imaging techniques and mathematical modeling. The effect of W-DeepLab network-assisted diagnosis of images under white light was analyzed, and the value of Narrow Band Imaging and Blue Laser Imaging in the diagnosis of early gastric cancer was compared. Because Blue Laser Imaging endoscopy can clearly observe the demarcation line and microvascular morphology; but when using Narrow Band Imaging observation, part of the demarcation line and microvascular morphology is not observed. The results show that Blue Laser Imaging is brighter than Narrow Band Imaging's endoscopic images, and it is easier to observe the microstructure of lesions under endoscopy, so as to accurately determine the nature of lesions.

## 1. Introduction

Gastric cancer originates from a malignant tumor of the gastric epithelium and is the second leading cause of cancer death in the world. There are large differences in the incidence of gastric cancer in countries and regions around the world [1]. Early gastric cancer usually does not have any symptoms, and even if there is, it may be caused by the combination of atrophic gastritisaQ, Helicobacter pylori infection, or functional dyspepsiaa, rather than the early gastric cancer lesions themselves. When there are alarm symptoms such as aggravation of abdominal symptoms, anorexia, weight loss, anemia, and melena, most of them are advanced gastric cancer. The overall prognosis of gastric cancer in my country is poor. Because the lesions of early gastric cancer are often small, it is difficult to diagnose early gastric cancer by regular gastroscopy. Endoscopic narrow-band imaging technology and staining technology make the gastric mucosal gland openings and microvessels of the lesions more clearly displayed under the microscope by changing the spectral and chemical staining methods, respectively, and it is easier to identify gastric cancer lesions [2, 3]. A mathematical model is an abstract description of a problem using systematic symbols and mathematical expressions. Mathematical modeling can be seen as the process of transforming a problem definition into a mathematical model. Medical imaging technology and mathematical modeling can effectively help the efficiency of early gastric cancer diagnosis.

My country is a country with a high incidence of gastric cancer. Most of the patients are in the middle and late stages when they go to the clinic. Even if they receive surgical treatment, the survival rate and quality of life are not ideal [4]. Klimenko A A presents the most common and clinically convenient classification and staging system for gastric cancer, confirming the need for the earliest possible diagnosis and verification of the stage of the tumor process. Modern methods of gastric cancer diagnosis are considered in detail, including esophagogastroduodenoscopy (EGD) as the method of choice for the initial detection of gastric cancer, and various radiographic modalities, including multi-spiral computed tomography and endoscopic ultrasonography (EUS), combined with chromoendoscopy, narrow-band tomography, and confocal laser endoscopy [5]. Mikhaleva LM reviewed mixed gastric cancer. Compared with other types, mixed gastric cancer has the characteristics of older patients (over 65 years old), larger tumors, obvious local tumor infiltration, and high metastasis rate. Further in-depth studies of mixed-type gastric cancer in the context of its morphological histological tumor components, as well as tumorigenesis mechanisms, are warranted as they may aid in the early diagnosis of tumors and more accurate prediction of outcome and selection of appropriate management strategies, i.e., determination of the extent of surgical manipulation and further medical treatment, taking into account the molecular characteristics of the tumor and its PD-L1 status, will significantly affect the 5-year survival rate of the patient in the long run [6]. In Kumar S's study, annual endoscopic surveillance via the Cambridge protocol was recommended for patients with delayed surgery, including biopsy of any lesions and at least 30 random biopsies from the antrum, transition zone [7]. Therefore, it is of practical significance to study the diagnosis of early gastric cancer based on medical imaging technology and mathematical modeling.

Common gastroscopy combined with pathological biopsy is the main basis for the selection of early gastric cancer diagnosis and diagnosis and treatment in my country. However, endoscopic biopsy samples are shallow and few, and the biopsy process is empirical, random, and blind. Whether the focal biopsy tissue can fully reflect the overall condition of the lesion is still controversial. This paper discusses the diagnostic ability of NBI-ME, gastroscopic biopsy, and W-DeepLab modeling for early gastric cancer, in order to provide some theoretical basis for the diagnosis of early gastric cancer.

## 2. Research on the Diagnosis of Early Gastric Cancer Based on Medical Imaging Technology and Mathematical Modeling

### 2.1. Medical Imaging Technology

#### 2.1.1. Blue Laser Imaging (BLI)

BLI is a new generation of IEE for the LASEREO system, which uses lasers with two wavelengths of 410 and 450 nm as the light source [8]. As a new type of endoscope, BLI can more clearly observe the morphology of microvessels and microstructures on the surface of gastric mucosa, thereby helping to find lesions and improve the detection rate of early gastric cancer. In the BLI-bright observation mode, its bright field of view can make subtle observations of distant lesions, while in the ME-BLI mode, the microvascular pattern, microglandular pattern, and demarcation line of the lesion can be clearly observed display. Based on the diagnostic criteria of the VS classification system, compared with WLE, BLI can clearly display the lesion boundary and provide a more accurate diagnosis of EGC [9]. Although BLI has greatly improved the diagnostic accuracy of lesion boundaries, a combined study of BLI with other IEEs is still needed to further evaluate the value of its combined application in detecting gastric lesion boundaries [10].

#### 2.1.2. Narrow Band Imaging (NBI)

Based on the VS classification and diagnosis method, ME-NBI can clearly display the structure of microglandular blood vessels and microglandular ducts on the surface of gastric mucosa. Due to differences in EGC histology and background mucosal inflammation, in undifferentiated EGCs, the cancerous tissue is often not exposed to the lesion surface. However, NBI can only obtain a more accurate diagnosis of the depth of EGC infiltration in differentiated EGC, and further studies are needed to provide evidence for undifferentiated EGC [11, 12].

ME-NBI diagnostic criteria for early gastric cancer: ME-NBI subsurface microstructure (MS) definition includes crypt opening, marginal crypt epithelium, and the part between crypt openings; surface microvascular structure (MV) subepithelial capillaries, collections Veins, and pathological microvessels [13]. According to the microstructure and vascular morphology, MS and MV were divided into three types: regular, irregular, and absent. Regular microstructure, that is, the marginal crypt epithelium shows a uniform shape such as linear, elliptical, curved, annular, and other structures, with symmetrical distribution and regular arrangement; irregular surface microstructure, that is, showing irregular linear, curved, villous, and other structures, irregular in shape, various in structure, non-uniform in structure, asymmetric in distribution, and irregular in arrangement; missing microstructure, that is, no marginal crypt structure and white opaque shape can be seen under endoscopy substance. Similarly, for regular microvessels, mucosal capillaries show a uniform shape, closed loop, or open; for irregular microvascular structure, microvessels show open, closed loop, twisted, branched, and other shapes, with different shapes. Uniform, asymmetric distribution, and irregular arrangement; missing microvessels, manifested as the disappearance of microvascular structures, are replaced by white opaque substances [14, 15]. According to the “VS classification system,” early gastric cancer can be diagnosed if any of the following is satisfied; otherwise, it is a non-cancerous lesion: (1) irregular surface microstructure (IMSP) and clear demarcation line (DL); (2) irregular Microvessels (IMVP) and specific lines of differentiation (DL) [16].

### 2.2. W-DeepLab Modeling

Image segmentation is a critical step in image understanding. The basis of segmentation mainly includes (1) the segmented area is a homogeneous area, which can be grayscale, texture, or other specific features; (2) the interior of the area is smooth and free of small holes; (3) the boundaries of each area are complete, the space is complete, and the location normal, no cracks [17]; (4) there should be obvious differences between adjacent areas, and a unified judgment basis should be selected.

First, perform 4 times bilinear upsampling on the features extracted by the encoder and temporarily record this result as D1; then reduce the number of channels from the feature map D2′ extracted from DCNN with the same scale as D1 to obtain D2. It is obtained by 1 × 1 convolution with D1. The features of these scales usually have 512 or 256 channels in DCNN, but not so many feature channels are extracted by the encoder, so it is necessary to reduce the number of channels, if direct. If the connection is made without dimensionality reduction, the weight of D2′ will be increased invisibly, which will greatly increase the difficulty of network training; for the subsequent work of connecting D1 and D2, the result is first recorded as D3, and the features of D3 are fine-tuned. Do the normal operation of 3 × 3 convolution and finally perform 4 times upsampling operation to obtain the segmentation result [18].

In this paper, the W-DeepLab network uses the cross-entropy loss function to measure the difference between the model predicted value and the actual value.

When using logistic regression to solve the binary classification problem, the known samples have *m* labels, the training set [(*x*(1), *y*(1)), (*x*(2), *y*(2)), ⋯, (*x* (*m*), *y*(*m*))], and the definable cross-entropy loss function is derived from the maximum likelihood estimation combined with the logistic classifier as:

(1) $$\begin{array}{c} J\left(\theta \right)=‐\frac{1}{m}\left[\overset{m}{\underset{i=1}{\sum }}y^{\left(i\right)}\log h_{\theta }\left(x^{\left(i\right)}\right)+\left(1-y^{\left(i\right)}\right)\log\left(1-h_{\theta }\left(x^{\left(i\right)}\right)\right)\right], \end{array}$$

where *h*_*θ*_(*x*) is the predicted or activation value.

The original loss function is denoted by *C*_0_, and the loss function after weight decay is applied to the parameter *w* is:

(2) $$\begin{array}{c} C=C_{0}+\frac{\lambda }{2n}\underset{w}{\sum }w^{2}. \end{array}$$

The regularization coefficient is denoted as *λ*, and in this paper, *λ*=0.00004, and the number of samples is denoted as *n*. Taking the derivation of the parameter *w* in the formula, the formula can be obtained:

(3) $$\begin{array}{c} \frac{\partial C}{\partial w}=\frac{\partial C_{0}}{\partial w}+\frac{\lambda }{n}w. \end{array}$$

The learning rate is represented by *η*, and weight decay is added during training. At this time, the formula of the parameter *w* is updated to:

(4) $$\begin{array}{c} w⟶w-\eta \frac{\partial C_{0}}{\partial w}-\frac{\eta \lambda }{n}w=\left(1-\frac{\eta \lambda }{n}\right)w-\eta \frac{\partial C_{0}}{\partial w}. \end{array}$$

In the above formula, 1 − *ηλ*/*n* is a coefficient less than 1, and its function is to reduce the value of *w*. A lower network complexity model will also fit the data better.

## 3. Investigation and Research on the Diagnosis of Early Gastric Cancer Based on Medical Imaging Technology and Mathematical Modeling

### 3.1. Research Objects

Select patients who have undergone electronic gastroscopic examinations in M Hospital from 2020 to 2021, and the nurses in the endoscopy room will number the patients in the order in which the patients made gastroscopy appointments, starting from the first patient who underwent gastroscopy on January 1, 2020; the number starts from the 1st and records the patient's name, age, gender, clinical symptoms, initial diagnosis, and contact information. According to the number, the odd-numbered patients were treated as the control group for white light endoscopy and NBI examination, and the even-numbered patients were used as the experimental group for white light endoscopy and BLI examination. The numbering nurse in the endoscopy room just numbers and does not know the grouping situation.

Inclusion criteria: (1) Patients who signed informed consent. (2) No serious infection. Exclusion criteria: (1) Patients with mental illness and severe heart failure. (2) Patients with a history of abdominal surgery and mucosal structures cannot be observed. (3) Patients with acute upper gastrointestinal bleeding, gastric perforation, or upper gastrointestinal obstruction. According to the inclusion and exclusion criteria, a total of 4040 people were included in this study, of which 1864 people in the control group were observed by NBI endoscopy; 2176 people in the experimental group were observed by BLI endoscopy.

### 3.2. Endoscopy Procedure

Choose from the GIF-H260ZNBI endoscope and the EG-L590WR blue laser endoscope. Patients undergoing gastroscopy are given an empty stomach on the day of the examination, and the oropharynx is administered local anesthesia with mucus prior to the examination. The control group underwent NBI examination, and the experimental group underwent BLI endoscopy. The control group underwent white light endoscopy to obtain clear images of the lesions. Then, after finding the lesion, switch to NBI mode to further observe the shape, boundary, and microstructure of the lesion, and make an endoscopic diagnosis. Finally, 3-5 pieces of mucosal tissue are taken from the edge of the lesion and sent for pathological biopsy. The endoscopic observation of BLI lesions in the experimental group generally adopted the following methods: first, clear images of the lesions were obtained through white light endoscopy, and the color and microscopic structure of blood vessels on the surface of the lesions were observed. After the lesions were detected, the BLI-light mode was used to observe and further analyze the histological properties of the lesions. Make a judgment, and finally use the BLI function to observe the muscle tissue and wound structure in a large picture, and make an endoscopic diagnosis of the wound. Finally, 3-5 pieces of mucosal tissue were taken at the edge of the lesion and sent for pathological biopsy.

### 3.3. Model Training

The ordinary white light endoscopic images studied in this paper have only 100 valid raw data before augmentation, and a new network can hardly be trained in the case of scarce data resources. Therefore, fine-tune is only performed when the parameters are initialized. In the shallow feature extraction, the existing data model is fine-tuned by combining the characteristics of ordinary white light endoscopic image data, as shown in Figure 1.

This paper proposes the W-DeepLab network for computer-aided diagnosis of intestinal metaplasia and trains it using a white light endoscopic image dataset. The dataset is randomly divided into three parts, namely, training set, validation set, and test set. The training system corresponds to the model parameters, the verification system adjusts the hyperparameters of the model, and the test system is used to evaluate performance, and the test system does not participate in model training and verification. This article uses the TensorFlow1.6.0 deep learning framework and the Python language program version 3.5.2 for testing. The initial learning rate is 0.0001, and the learning rate decreases according to the curve as the number of iterations increases.

## 4. Analysis and Research on the Diagnosis of Early Gastric Cancer Based on Medical Imaging Technology and Mathematical Modeling

### 4.1. Gender Composition of the Two Groups of Subjects

There were 2176 cases in the experimental group, 52% male and 48% female, and 1864 cases in the control group, as shown in Figure 2. There were 38 men and 62 women, respectively. The Pearson *χ*^2^ test was performed on the gender of the two groups of research subjects, and there was no statistical difference in the gender composition of the two groups of subjects, as shown in Table 1.

### 4.2. Experimental Results of Images under White Light

The segmentation speed of FCN-32s, DeepLabv3+, and W-DeepLab was tested to enable a more comprehensive assessment of the computer-aided diagnosis network for intestinal metaplasia. The test results of each evaluation index of each network on the ordinary white light endoscopy image dataset are shown in Table 2. The better the performance of the network, the higher the specificity and sensitivity will be. From the test results, it can be clearly concluded that the specificity and sensitivity of the W-DeepLab network are better than other network models, reaching 97% and 91%, respectively, and the MIoU value of the W-DeepLab network is also the highest. The best is 88%, which is significantly higher than 62% of FCN-32s and 77% of DeepLabv3+. The most important thing is that the W-DeepLab network is as high as 98% in terms of global pixel accuracy, which is significantly better than the other two networks, as shown in Figure 3.

In the classification task of medical images, the classification accuracy is usually evaluated by the characteristic curve (ROC) index. The area enclosed by the ROC curve and the horizontal axis is called AUC. The better the classification method, the greater the AUC value. By entering the AUC value into the measurement network, the standard is to make the verification of the network proposed in this paper more comprehensive and objective. The AUC values of different models are shown in Table 3. The AUC value of the W-DeepLab network is 0.98, which is much larger than the 0.88 of FCN-32 s and 0.91 of DeepLabv3+. These experiments are enough to fully demonstrate that the W-DeepLab network can make a positive contribution to the computer-aided diagnosis of intestinal metaplasia.

### 4.3. Comparison of the Value of NBI and BLI in the Diagnosis of Early Gastric Cancer

Irregular microvascular morphology and irregular surface microstructure with demarcation lines were observed under endoscopy, which can be diagnosed as early gastric cancer. For early gastric cancer, among 1864 patients in the control group, 178 were diagnosed with early gastric cancer by NBI endoscopy. Compared with the early gastric cancer diagnosed by the pathology department, 204 patients were diagnosed by endoscopy, which was consistent with the results reported by the pathology department.

Among the 2176 patients in the experimental group, 211 patients were diagnosed with early gastric cancer by BLI endoscopy. Compared with the early gastric cancer diagnosed by the pathology department, the endoscopic diagnosis of 191 patients was consistent with the pathological report, and 7 patients were diagnosed with early gastric cancer.

The chi-square test was used to calculate the difference in sensitivity and specificity of NBI and BLI for the diagnosis of early gastric cancer, as shown in Table 4. The difference in sensitivity (*P* = 0.021) between the two was calculated to be statistically significant, while the difference in specificity (*P* = 0.409) between the two was not statistically significant, as shown in Figure 4.

## 5. Conclusions

The timely detection of early gastric cancer has become the key to whether patients can receive early treatment. Therefore, improving the diagnosis level of early gastric cancer will significantly reduce the mortality of gastric cancer and improve the quality of life of patients. This study compared the value of NBI and BLI in the diagnosis of early gastric cancer, but the specificity of the two was not statistically significant. All patients with correct diagnosis of early gastric cancer in the NBI picture had significant IMVP and DL or IMSP and DL. However, in 13 benign LGIN lesions, these three major structures failed NBI endoscopy. The doctor's understanding of early gastric cancer and the experience of endoscopic surgery often determine the direction of diagnosis. The missed diagnosis was due to the fact that the mucosal surface was covered with “white substances”, which affected the judgment of microvessels and microstructures. Later, the images were checked and corrected to early gastric cancer. This paper also introduces the related experiments of applying W-DeepLab network in computer-aided diagnosis of intestinal metaplasia. The ordinary white light endoscopic image was selected as the image used in the data set, and then the raw data of the ordinary white light endoscopic image obtained from the Department of Gastroenterology of the First Affiliated Hospital were processed into data that could be recognized by the semantic segmentation network. It also introduces several mainstream indicators for evaluating computer-aided diagnosis ability and methods for optimizing model training; finally, the models are tested and compared on the white light endoscopy image test set. The research results show that the computer-aided diagnosis technology for intestinal metaplasia based on the W-DeepLab network has the best effect; and in the comparison between the W-DeepLab network and other semantic segmentation networks, the AUC value, specificity and sensitivity, etc. properties all perform better.

The study also had some limitations. First, this study is a single-center retrospective study, which may have limitations in case selection and cannot fully cover all cases. Therefore, further verification with more cases is required. Second, endoscopic diagnostic results are not completed by the same physician, and different levels of clinical experience may affect the accuracy of endoscopic results. Finally, the diagnostic ability of BLI endoscopic mucosal microstructure typing on the differentiation degree of EGC was not further analyzed in this study, and further research is needed to determine in the future.

## Figures and Tables

**Figure 1:** The fine-tune method initializes network parameters.

**Figure 2:** Male to female ratio.

**Figure 3:** Model experimental results in the testing phase of the white light endoscopic image dataset.

**Figure 4:** Results of the chi-square test.

**Table 1:** Gender distribution of the two groups of subjects.

Grouping	Test group (%)	Control group (%)	*P* value
Male	52	38	0.42
Female	48	62	
Total	100	100	

**Table 2:** Test results of each evaluation index.

Model	Accuracy	Sensitivity	Specificity	MIoU	Time
W-DeepLab	98%	91%	97%	88%	10frame/s
DeepLabv3+	80%	78%	93%	77%	12frame/s
FCN-32s	81%	70%	85%	62%	2frame/s

**Table 3:** AUC values for different models.

Model	W-DeepLab	DeepLabv3+	FCN-32s
AUC	98%	91%	88%

**Table 4:** Comparison of the value of NBI and BLI in the diagnosis of early gastric cancer.

Group	Sensitivity	Specificity
NBI	79%	92%
BLI	90%	98%
P	0.018	0.44

## Data Availability

The data underlying the results presented in the study are available within the manuscript.
